# Intervention of the Syndrome-Position Point Selection Method on Idiopathic Tinnitus of Phlegm-Fire Stagnation Pattern: A Randomized Controlled Study

**DOI:** 10.1155/2022/9664078

**Published:** 2022-03-23

**Authors:** Qiang Su, Xin Shi, Jianning Zhang, Ming Li

**Affiliations:** ^1^Department of Rehabilitation Medicine, The Second Affiliated Hospital of Bengbu Medical College, Bengbu City 233000, Anhui Province, China; ^2^Department of Medicine, Hangzhou Normal University, Hangzhou City 311121, Zhejiang Province, China; ^3^Department of Otolaryngology, Yueyang Integrated Traditional Chinese and Western Medicine Hospital Affiliated to Shanghai University of Traditional Chinese Medicine, Shanghai City 200437, China

## Abstract

**Objective:**

To investigate the clinical effect of the syndrome-position point selection method on the intervention of idiopathic tinnitus of the phlegm-fire stagnation pattern.

**Methods:**

One hundred patients with idiopathic tinnitus of phlegm-fire stagnation pattern who met the inclusion criteria were randomized into the treatment group and the control group by the random number table method, with 50 cases in each group. The treatment group (syndrome-position point selection method) was treated with acupuncture at the corresponding acupoints for tinnitus and associated symptoms and the corresponding acupoints located in Wernicke's area of scalp projection, while the control group (traditional acupuncture method) was treated with the combination of acupuncture points with the most frequent occurrence in the tinnitus research literature for acupuncture treatment. Both groups received acupuncture twice a week for 5 weeks. The efficacy was evaluated before and after treatment with the Tinnitus Severity Inventory (TSI), Sleep Spiegel Questionnaire, Self-Rating Anxiety Scale (SAS), and Self-Rating Depression Scale (SDS).

**Results:**

The 100 patients with idiopathic tinnitus of phlegm-fire stagnation pattern completed 5 weeks of clinical treatment and a month of follow-up with no loss of patients and no adverse event reports. Three patients recovered with the disappearance of the tinnitus symptoms in the treatment group after 5 weeks of treatment. After 5 weeks of treatment, obvious differences between the two groups were observed in the TSI scores (*P* < 0.05) and the Spiegel scores, with a better Spiegel score in the treatment group than in the control group (*P* < 0.05). Compared with the control group, the depression (SDS score) and anxiety (SAS score) of tinnitus patients in the treatment group were markedly improved (*P* < 0.05).

**Conclusion:**

In line with the principle of symptomatic treatment and based on the modern imaging data, the syndrome-position point selection method is more accurate and effective compared with the traditional acupoint selection method, which significantly improves the symptoms, sleep quality, and psychological state of patients with idiopathic tinnitus of the phlegm-fire stagnation pattern.

## 1. Introduction

Idiopathic tinnitus is defined as a subjective symptom of patients with the perception of sound in their ear or head without a sound source or electrical stimulation in the surrounding environment, often with or without adverse psychological reactions such as hearing loss, sleep disorders, impatience, inability to concentrate, and anxiety. Due to its complex etiology, no specific drugs have been found to completely treat it [1–4]. Although the disease has a certain self-healing rate, patients should not wait passively. The etiology should be clarified as far as possible, and a targeted treatment method should be selected in clinical treatment [5, 6]. Over the years, Chinese traditional dialectical medicine has made many research achievements in tinnitus treatment, among which acupuncture therapy is one of the important methods. Acupuncture is an important branch of traditional Chinese medicine (TCM) and its acupoint selection theory has been practiced in previous research results, which can hardly reflect the characteristics and advantages of the acupuncture dialectical system theory in clinical treatment, thus leading to an unsatisfactory therapeutic effect. Considering the fundamental purpose of acupuncture treatment, only the effective combination of disease, symptoms, and positions can ensure the final therapeutic effect. The New England Journal of Medicine [7] reported that tinnitus could be inhibited by repeated stimulation of implanted electrodes, and positron emission tomography (PET) showed nerve activation in the posterior part of the right superior temporal gyrus, supramarginal gyrus, and right superior temporal sulcus. The whole-brain PET-CT detection of patients with idiopathic tinnitus shows no significant hypermetabolism of glucose in the bilateral auditory cortex and visual cortex under the condition of visual and auditory opening, but hypermetabolism of glucose in the left Wernicke area. Therefore, the scalp projection data in the Wernicke area has a high guiding value for the acupuncture treatment of patients. Phlegm-fire stagnation pattern is a common disease type in TCM syndrome differentiation and treatment of tinnitus. Therefore, this paper advocates to formulate a new acupuncture point selection scheme for tinnitus treatment based on the symptoms of patients with tinnitus imaging data (Wernicke scalp projection), that is, the syndrome-position point selection method, and further explores the intervention effect of the method on idiopathic tinnitus of the phlegm-fire stagnation pattern, so as to improve the clinical efficacy.

## 2. Materials and Methods

### 2.1. Research Subjects

The inclusion criteria are as follows: (1) patients met the clinical diagnostic criteria of idiopathic tinnitus and the diagnostic criteria of idiopathic tinnitus with phlegm-fire stagnation pattern in the *Otolaryngology of Traditional Chinese Medicine* [8]; (2) patients had clear complaints, with complete clinical data and no expression disorders; (3) the course of disease did not exceed 24 months; and (4) patients and their families were informed of and agreed to this study.

The exclusion criteria are as follows: (1) patients with tinnitus caused by congenital defects, tumors, trauma, or other diseases; (2) women during pregnancy or lactation; (3) patients complicated with other serious physical diseases or bleeding tendency; (4) patients with low treatment compliance or quitting halfway; and (5) patients with severe psychological anxiety or depression.

One hundred patients with idiopathic tinnitus of phlegm-fire stagnation pattern who were treated at the Tinnitus Center of Yueyang Hospital of Integrated Traditional Chinese and Western Medicine affiliated to Shanghai University of Traditional Chinese Medicine from June 2011 to January 2013 were selected as the research subjects. The study was approved by the hospital ethics committee and was conducted in accordance with the Declaration of Helsinki (as revised in 2013) [9].

### 2.2. Grouping and Treatment Plans

One hundred patients with idiopathic tinnitus of phlegm-fire stagnation pattern who met the inclusion criteria were randomized into the treatment group (syndrome-position point selection method) and the control group (traditional acupuncture method) by the random number table method, with 50 cases in each group. Both groups received acupuncture twice a week for 5 weeks..

1. Acupuncture methods. After the selection of acupoints and routine disinfection of hands, the acupuncturist used both hands to puncture with the nail pressing needle inserting method according to the characteristics of the acupoint positions. The direction and depth of acupuncture were strictly in accordance with the requirements of acupuncture manipulation. After needle insertion, twisting, lifting, and thrusting, and the reducing method were performed, with lifting and thrusting between 0.3 and 0.5 cm, and twisting around 180° at a frequency of 50–60 cycles/min. Besides, they were performed with the same amplitude and frequency until adequate Qi was obtained. The needles were left for 30 minutes with no manipulation during needle retention. For the withdrawal of the needles, the left thumb and index finger were used to hold the sterilized dry cotton ball and gently press on the acupuncture points, while the right hand held the needles for slight twirling, slowly lifted the needles to the subcutaneous tissue, stayed for a moment, and then slowly withdrew the needles. After withdrawal, the pinholes were not pressed unless bleeding occurred. In the treatment group, the electroacupuncture apparatus had a set of positive electrodes connected at the Shuaigu point of the affected side and a set of negative electrodes connected at the Tinggong point of the affected side. In the control group, the electroacupuncture apparatus had a set of positive electrodes connected at the Yifeng point of the affected side and a set of negative electrodes connected at the Tinggong point of the affected side. A continuous wave of 2 Hz was selected as the stimulation frequency and waveform, and the current intensity was gradually increased starting from 0 mA according to patients' tolerance. After 30 min, the output potentiator was withdrawn to the 0 position, the switch was turned off, the lead was removed, and then the needle was removed with the needle withdrawal method, as shown in Table 1 and Figure 1 for specific points.
2. Needles. Huatuo 0.25 × 25 mm disposable acupuncture needles and Huatuo G6805-2 low frequency electronic pulse therapeutic apparatus (Suzhou Medical Supplies Factory), with a frequency of 50/60 Hz and an input power of 10VA.

### 2.3. Observation Indexes

The condition improvement, sleep quality, and psychological state of the patients with idiopathic tinnitus of phlegm-fire stagnation pattern in both groups were evaluated before and after treatment with the Tinnitus Severity Inventory (TSI) [10], Sleep Spiegel Questionnaire [1], Self-Rating Anxiety Scale (SAS) [11], and Self-Rating Depression Scale (SDS) [12]. TSI is an internationally recognized tinnitus assessment scale with a total of 25 items, including the environment of tinnitus, duration of tinnitus, the impact of tinnitus on sleep, the impact of tinnitus on study and work, tinnitus-caused restlessness, and patients' overall feeling of tinnitus.

### 2.4. Efficacy Evaluation

In this study, the single-blind method was adopted, and the outpatient doctors who were not involved in grouping and treatment observed, recorded, and evaluated the patients' treatment compliance and clinical response related to treatment. Experts who did not participate in grouping and treatment were arranged to check each evaluation form.

### 2.5. Statistical Treatment

The software SPSS17.0 for windows was used for statistical analysis. All the measurement data were expressed as (‾*x* ± *s*), with the test level of *α* = 0.05. The enumeration data were tested by X^2^. The data consistent with normality and homogeneity of variance were statistically assessed by the *t*-test for paired data before and after treatment in each group, and the comparison among groups was assessed by ANOVA or *t*-test. The rank-sum test was used for data that did not meet normality and homogeneity of variance.

## 3. Results

Tinnitus is a chronic recurrent disease. The patients were followed up 1 month after treatment. The baseline data and sociodemographic characteristics of both groups were similar at the time of examination (*P* > 0.05), as shown in Table 2. The 100 patients with idiopathic tinnitus of phlegm-fire stagnation pattern completed 5 weeks of clinical treatment and a month of follow-up with no loss of patients and no adverse event reports. Three patients recovered with the disappearance of the tinnitus symptoms in the treatment group after 5 weeks of treatment. After 5 weeks of treatment, obvious differences between the two groups were observed in the TSI scores (*P* < 0.05) and the Spiegel scores, with a better Spiegel score in the treatment group than in the control group (*P* < 0.05). Compared with the control group, the depression (SDS score) and anxiety (SAS score) of tinnitus patients in the treatment group were markedly improved (*P* < 0.05; Figure 2).

## 4. Discussion

The traditional acupoint selection method believes that the acupoints of Tinggong, Tinghui, and Yifeng are the most frequently used acupoints in the treatment of tinnitus in the ancient literature. The treatment purpose is to dredge qi and blood from the meridians of the ears, assist in the transportation of heart and kidney, and thus achieve the effect of eliminating tinnitus. The acupoint selection scheme can accelerate the microcirculation of the inner ear by stimulating the acupoints. However, the effect is obvious but erratic, with many patients complaining of recurrence of the disease after treatment [13–15]. Since ancient Chinese medicine believes one prescription is for one person, one point should correspond to one person in acupuncture treatment of tinnitus. Clinically, closely related to hemorheology, tinnitus is often accompanied by abnormal hemorheology, resulting in slow or stagnant blood flow in the local tissue of the cochlea. Besides, hemorheology changes caused by different symptoms also vary. Therefore, the selection of acupuncture points for tinnitus needs to be carried out dialectically according to the specific syndromes of tinnitus [16–18]. Based on the understanding of idiopathic tinnitus with a phlegm-fire stagnation pattern in both Chinese and Western medicine, this study aimed to innovate the acupoint selection scheme. On the basis of conventional and dialectical acupoint selection combined with the imaging results of tinnitus, this study carried out the local acupoint selection through the imaging manifestations in the Wernicke area of the cerebral cortex and performed the syndrome-position point selection according to the imaging features of the adverse tinnitus symptoms. Therefore, in the treatment group, this study selected Tinggong point in the traditional scheme to dredge qi and blood from the meridians of the ears, Shuaigu and Tianchong in the Wernicke projection area to inhibit glucose metabolism, Baihui, Shenmen, and Anmian to improve the sleep of patients, and Siguan to reduce adverse conditions such as anxiety and depression. Compatibility of the acupoints, one qi and one blood, one yang and one yin, and one ascending and one descending, has a synergistic effect, which could clear heat, promote diuresis, activate meridians, resolve phlegm, soothe the liver-gallbladder, and resolve stagnation for tranquilization. Besides, the addition of Fenglong could eliminate phlegm and dredge meridians.

### 4.1. Theoretical Basis and Material Basis of the Syndrome-Position Point Selection Method

This study believes that idiopathic tinnitus is an abnormal nerve impulse that is not uploaded in normal sound coding, and its central sensory cortex may be located in the Wernicke area. Therefore, PET-CT imaging results of the Wernicke area are the material basis of the syndrome-position point selection method. Therefore, in accordance with the principle of “treating where the meridians pass,” the corresponding acupoints of scalp projection in this region were selected, and the characteristic acupoints for treating sleep disorders and psychological discomfort were selected to group acupoints. Specifically, on the basis of the traditional acupoint selection method for tinnitus, Shuaigu and Tianchong in the scalp projection area of the Wernicke area, Baihui, Shenmen, and Anmian for improving sleep, and Siguan for improving anxiety and depression, were combined to form a new acupoint selection scheme, that is, the syndrome-position point selection method.

Traditional Chinese medicine (TCM) believes that tinnitus mainly results from deficiency and excess, in which the former is caused by a deficiency of qi and the blood of the internal organs, while the latter is due to six exogenous pathogenic factors, phlegm stasis, and the disturbance of excess fire. Therefore, most scholars believe that the principle of TCM treatment for tinnitus should be based on overall conditioning and syndrome differentiation and treatment, which not only starts from the adjustment of the overall balance of viscera, and yin and yang, but also needs to combine dredging and tonifying to regulate qi [19–21]. The theoretical basis of scalp acupuncture has been described in many ancient books. *Miraculous Pivot and Great Confusion Theory* [22] states that the essence of internal organs in the body infusing upward into the eyes enables people to see things clearly, which forms the eye system combining with the meridians. The system is connected upward to the bran and backward to the middle of the nape. *Plain questions - Refined Theory of Meridians* [23] demonstrates that the governor meridian goes up to Fengfu, enters the brain, goes up to the top, follows the forehead, and reaches the nasal bridge. In the six yin meridians of hand and foot, the Heart Meridian of Hand-shaoyin goes up to the pharynx and connects the eye system, and the Jueyin liver meridian of foot goes up and meets the governor meridian in the head, while other yin meridians directly go up to the head after passing through the Yang meridians in the head. The head (brain) is the capital of the Qingyang and the marrow sea, which is the house of mental activity, the dominating power mastering the functional activities of internal organs and meridians, and an important part of regulating qi and blood throughout the whole body. The abovementioned scriptures fully illustrate that the head is closely related to the internal organs and meridians, which is the theoretical basis of scalp acupuncture in treating diseases in TCM.

In this study, the 100 patients with idiopathic tinnitus of phlegm-fire stagnation pattern completed 5 weeks of clinical treatment and a month of follow-up with no loss of patients and no adverse event reports. Three patients recovered with the disappearance of the tinnitus symptoms in the treatment group after 5 weeks of treatment. After 5 weeks of treatment, obvious differences between the two groups were observed in the TSI scores (*P* < 0.05). These results were consistent with the study of Ihsan Kuzucu [24], demonstrating that the syndrome-position point selection method can significantly alleviate the clinical symptoms and improve the curative effect of patients with idiopathic tinnitus of the phlegm-fire stagnation pattern.

### 4.2. Advantages of Acupuncture in Improving Sleep and Emotional Disorders of Tinnitus Patients

After 5 weeks of treatment, an obvious difference in the Spiegel scores was observed between the two groups, with a better score in the treatment group than in the control group (*P* < 0.05). Compared with the control group, the depression (SDS score) and anxiety (SAS score) of tinnitus patients in the treatment group were markedly improved (*P* < 0.05). The primary goals of clinical tinnitus treatment are to reduce or eliminate tinnitus symptoms directly, and then to alleviate the accompanying symptoms such as sleep disorders and psychological discomfort caused by tinnitus. According to various ancient medical books and modern clinical reports, acupuncture therapy is effective in alleviating adverse psychological reactions such as sleep disorders, anxiety, and depression, with definite and excellent long-term curative effects. This study further confirmed that acupuncture therapy based on the syndrome-position point selection method can effectively improve sleep and emotional disorders in patients with idiopathic tinnitus of the phlegm-fire stagnation pattern.

In conclusion, in line with the principle of symptomatic treatment and based on modern imaging data, the syndrome-position point selection method is more accurate and effective compared with the traditional acupoint selection method, which significantly improves the symptoms, sleep quality, and psychological state of patients with idiopathic tinnitus of phlegm-fire stagnation pattern. In addition, due to the limitations of modern imaging techniques such as fMRI, PET, and MEG, the promotion of this point selection method in dialectical tinnitus examination still needs further exploration and practice. For limited time and effort, this study only carried out clinical research on patients with idiopathic tinnitus of phlegm-fire stagnation pattern. Therefore, this topic still needs the collection of more research samples and data at different levels and dimensions to further explore the treatment methods for tinnitus and the role of effective methods in the whole treatment process.

## Figures and Tables

**Figure 1:** Selected acupoints. Note: ①Tinggong; ②Tinghui; ③Yifeng; ④Anmian; ⑤ Tianchong; ⑥ Baihui; ⑦Shuaigu; ⑧Hegu; ⑨Shenmen; ⑩Taichong; ⑪Fenglong.

**Figure 2:** Main effects and interactions in Tinnitus Severity Questionnaire (TSI), Spiegel questionnaire, self-rating depression scale (SDS), and self-rating anxiety scale (SAS) between groups at different times.

**Table 1:** Grouping and acupoint selection.

Group	Traditional acupoints	Additional acupoints	Dyssomnia	Anxiety and depression	Results of PET/CT detection
Treatment group	Tinggong (SI19)	Fenglong (ST40)	Baihui (GV20)	Hegu (LI4)	Shuaigu (GB8)
	Tinghui (GB2)		Anmian (EXTRA)	Taichong (LR3)	Tianchong (GB9)
	Yifeng (TE17)		Shenmen (HT7)		

Control group	Tinggong (SI19)	Fenglong (ST40)			
	Tinghui (GB2)				
	Yifeng (TE17)				

**Table 2:** Baseline data and sociodemographic characteristics of the patients.

Observation indexes	Treatment group	Control group	*t*/*X*^2^	P^△^
Gender (n)	Male = 24, Female = 26	Male = 21, Female = 29	0.364	0.546
Average age (years)	50.10 ± 16.11	47.40 ± 14.68	0.876	0.383
Duration of tinnitus (months)				
<3 months (n)	17 (34%)	25 (50%)	2.627	0.105
3–12 months (n)	19 (38%)	12 (24%)	2.291	0.130
>12 months (n)	14 (28%)	13 (26%)	0.051	0.822
TSI (points)	12.08 ± 3.62	11.84 ± 3.06	0.358	0.721
Spiegel (points)	17.28 ± 4.69	15.72 ± 3.94	1.801	0.075
SDS (points)	31.53 ± 5.95	31.55 ± 5.14	0.018	0.986
SAS (points)	31.25 ± 4.25	31.83 ± 4.13	0.692	0.491

*Note.* The values are the mean ± standard deviation. △Statistical significance was set at *P* < 0.05 using the one-way ANOVA.

TSI, Tinnitus Severity Inventory; Spiegel, Spiegel Questionnaire; SDS, Self-Rating Depression Scale; SAS, Self-Rating Anxiety Scale.

## Data Availability

The data to support the findings of this study are available on reasonable request from the corresponding author.
